# Evaluation and Optimization Design for Microclimate Comfort of Traditional Village Squares Based on Extension Correlation Function

**DOI:** 10.1155/2022/6106463

**Published:** 2022-07-05

**Authors:** Qiang Guo, Xinxing Liu

**Affiliations:** ^1^Pan Tianshou College of Architecture, Art and Design, Ningbo University, Ningbo, Zhejiang 315211, China; ^2^School of Architecture and Urban-Rural Planning, Qingdao University of Technology, Qingdao, Shandong 266033, China

## Abstract

The evaluation approaches for microclimate comfort in traditional villages often ignore the year-round impact and the impact from dynamic and static behaviors, as well as the composite impact of wind and heat environments. To solve the problem, this study presents an evaluation and optimization design strategy for microclimate comfort of traditional village squares based on extension correlation function, using field survey, computer simulation, and example analysis. Firstly, the wind and heat environments in the space of the square were measured on the site with an ultrasonic integrated weather station. Secondly, simulation parameters were configured on PHOENICS (computational fluid dynamics software), namely, boundary conditions, wind environment, heat environment, and green plants, and used to simulate the wind and heat environments in the space of the square, followed by a correlation analysis between the simulation results and the measured results. Finally, the extension correlation function was adopted to comprehensively evaluate the microclimate comfort of the preliminary design scheme, and the design scheme of the square was finalized through repeated adjustments. The proposed strategy was verified on an example: Xieduqi square, Zoumatang village, eastern China's Zhejiang Province. The example analysis shows that the proposed strategy is highly operable. The research effectively improves the optimization design of traditional village squares, extends the digital technology system of traditional villages, and greatly drives rural construction in the future.

## 1. Introduction

### 1.1. Research Review

Traditional Chinese villages, especially those in Jiangsu and Zhejiang, are often blessed with a superior landscape environment, a profound history, and a convenient road transport system, as well as well-established infrastructure and public service facilities. Thanks to numerous rural revitalization policies (e.g., the project of one thousand demonstration villages and rectification of ten thousand villages, the beautiful village initiative, and the future village initiative), and heavy government investments, traditional villages are constantly attracting a large population from urban areas, and poised to be ideal human settlements in future. In recent years, more and more attention has been paid to microclimate comfort in rural spaces. The precision control of microclimate can create an energy-efficient, environmentally friendly, ecological, and comfortable rural space, which will significantly promote the construction of future villages, and energize the sustainable development of villages.

Microclimate refers to the local climate formed by the influence of the underlying surface. The comfort of microclimate, which can be measured by body comfort, is the satisfactory state of humans in a small-scale climate environment [22]. Microclimate comfort mainly consists of wind comfort and heat comfort. Most of the existing studies have adopted the Beaufort wind comfort criteria and heat comfort criteria, focusing on one of the two comforts. For example, many scholars explored the influence of greening methods (green space, tree arrangement, urban form, street form, and architectural form) over microclimate comfort of the square [1–7, 23]. Some scholars verified the heat comfort in the microclimate of the semiclosed courtyard space through numerical simulation [8, 9]. Soflaei et al. [24] adjusted the microclimate comfort of traditional Iranian courtyards, in the light of direction, size, and proportion. Tumini et al. [10] presented an urban renovation design strategy based on the modeling technology of microclimate heat comfort. Contraposing two typical urban spaces (squares and courtyards), Chatzidimitriou and Yannas [11] explained the influence of geometry, landscape elements, and material properties over the heat comfort of pedestrians. Through quantitative simulation, generation, and optimization operations, Qiu and Yu [12] put forward a spatial form design method for urban squares based on the universal thermal climate index (UTCI). Huang [13] improved the Beaufort scale combined with the dynamic and static behaviors on squares, and proposed a way to optimize the spatial form of square space. Yan et al. [14] expounded on the principles and evaluation indices of human heat comfort, and established a human heat adaptation model based on the analysis method for heat comfort data, the dry, humid, and hot climate effects, and the environmental regulation. To sum up, the existing studies have overlooked the year-round impact (e.g., the typical weather days in winter and summer are considered, instead of simulating the climate around the year), the impact from user behaviors (e.g., the obvious difference between dynamic and static behaviors in the adaptability to wind and heat environments), and the composite impact of wind and heat environments on human comfort (e.g., wind is merely treated as an index of heat comfort evaluation, without further deliberation: the wind velocity should not surpass 5 m/s at the height of 1.5 m). Most of spontaneous human activities have difficulty to proceed in an uncomfortable environment. The frequency and quality of public activities are significantly affected by wind velocity, temperature, and humidity. Some of the recent reviews in the field of microclimate comfort are collated in Table 1 to initiate the discussions on a comprehensive perspective.

### 1.2. Problem-Solving Ideas

Wind and heat environments have a composite influence on human comfort [15]. For the wind and heat comfort of traditional villages, there is not yet a clear definition of the boundaries, or a composite evaluation method, making it impossible to realize the optimization design of the public space. Therefore, it is crucial to establish a composite evaluation strategy for the wind and heat comfort in the public space of traditional villages, considering the impacts from year-round climate, and static, and dynamic behaviors. The extension correlation function provides an innovative tool for developing such a strategy. The function can objectively quantify the degree for an element in the domain of discourse to have a certain attribute, and illustrate the quantitative change and qualitative change of these elements. Yang and Cai [25] developed multiple calculation methods for correlation functions. Among them, the standard domain, transition domain, and zero boundary are suitable for simulating the year-round climate, and the composite correlation function is very fit for evaluating wind and heat comfort comprehensively. Therefore, this study presents an evaluation and optimization design strategy for microclimate comfort of traditional village squares based on extension correlation function, using field survey, computer simulation, and example analysis. The research comprehensively considers year-round climate simulation, comprehensive evaluation of wind and heat comfort, and dynamic and static behaviors, breaks through industry technology barriers, and extends the digital technology system of traditional villages.

The remainder of this paper is mainly divided into methodology explanation, and case analysis. Methodology explanation describes the basic principles, detailed steps and precautions of measurement, simulation and optimal design of micro-climate comfort, in order to provide theoretical support for case analysis. Case analysis takes the Xieduqi square as an example to verify the effectiveness of the above methods more intuitively and concretely.

## 2. Methodology Explanation

The evaluation and optimization design for microclimate comfort of traditional village squares based on extension correlation function make full use of digital technologies like oblique photography, panoramic shooting, and information modeling, and generate the optimization design scheme for traditional village squares through the following steps: field measurement of wind and heat environments, simulation of wind and heat environments, preliminary design of microclimate comfort, and composite evaluation of microclimate comfort. The proposed strategy consists of three modules: field measurement of wind and heat environments (Module 1), simulation of wind and heat environments (Module 2), and composite evaluation and optimization design of microclimate (Module 3). Module 1 measures the wind and heat environments in the space of the target square on the site with ultrasonic integrated weather stations. Module 2 configures simulation parameters, such as boundary conditions, wind environment, heat environment, and green plants, on PHOENICS, simulates the wind and heat environments in the space of the square, and tests the correlations between measured results and simulation results. Module 3 employs the extension correlation function to comprehensively evaluate the microclimate comfort of the preliminary design scheme and finalize the scheme through repeated adjustments (Figure 1).

### 2.1. Measurement of Wind and Heat Environments

#### 2.1.1. Measurement Time, Locations, and Instruments

In a traditional village, the square is a large, regular shaped, frequently used, and highly open venue, which provides an important space for villagers to carry out public activities and handle public affairs. The microclimate comfort of the square is mainly affected by wind direction, wind velocity, air temperature, relative humidity, and solar radiation [26, 27]. To identify the problems of local microclimate, the field measurement of wind and heat environments should be performed on the typical weather days in winter and summer, when the wind is relatively heavy (greater than force 5), and the solar radiation is in place.

The measurement locations should be selected by three principles. (1) The balanced distribution of wind velocity: the instruments should cover the typical space as uniformly as possible, and avoid spaces that are highly occluded or enclosed. (2) The diversity of people flows and activities: the instruments should cover as many static and dynamic behaviors in the public space as possible. (3) The reasonability of the number of instruments: the measuring points should be arranged based on the number of available instruments, and at least meet the basic needs of measurement.

Considering the slow velocity and changeable direction of wind in traditional villages, this study chooses an ultrasonic integrated weather station (RS-FSXCS-N01-1). Based on ultrasonic principles, the ultrasonic integrated weather station has no limit on the starting wind velocity, and supports 360° all-dimensional measurement. Coupled with solar charging, the instrument can record weather data (e.g., temperature and wind velocity) in the long term.  Table 2 lists the main technical parameters of the ultrasonic integrated weather station.  Figure 2 shows the cloud platform responsible for data collection and monitoring for the instrument.

#### 2.1.2. Collection of Hourly Climate Data

The climate data released by the state differ significantly from the actual climate parameters in the target village. The difference would severely suppress the simulation accuracy. This study places one ultrasonic integrated weather station at 1.5 m above the tallest building in the village, with no occlusions in the surroundings. The measurement at this point began at the same moment as the measuring points on the square. In recent years, outdoor activities, such as recreation, shopping, and cultural experience, have gradually increased on traditional village squares. During the measurement, we used a panoramic camera (Insta360 Pro 2) or another fisheye camera [16] to take photos or videos at each measuring point, which record the details about the space state and user behaviors.

### 2.2. Simulation of Wind and Heat Environments

#### 2.2.1. Selection of the Simulation Software

As for village modeling, drone oblique photography was combined with the ContextCapture modeling software to automatically synthesize an aerial model of the target traditional village (Figure 3) [17]. In addition, the information model of the traditional village (.rvt format) was generated semiautomatically, using the Revit software and its Dynamo plug-in (Figure 4).

The numerical simulation was performed on PHOENICS 2019, the first commercial software for computational fluid dynamics (CFD) and heat transfer. The FLAIR module of the software provides various turbulence models, multi-phase flow models, multi-fluid models, combustion models, and radiation models. Users can load these programs and models by a little programming. In addition, the software supports parallel computing, and offers diverse postprocessing tools. It is very suitable for simulating rural planning and design.

#### 2.2.2. Setting of Simulation Boundaries

The square is connected to other spaces in the traditional village. If the simulation boundaries are too large, the computing load would be too high. Under the premise of ensuring analysis accuracy, the top priority in wind and heat environment simulation is to properly set the simulation range of the object. The range is not the boundary conditions of the computational domain. Normally, the simulation range is bounded by the tall buildings, streets, and alleys around the square. The streets and alleys can be properly extended until the paths bend and form an enclosed space.

#### 2.2.3. Parameter Setting for Wind Environment

According to the requirements of POLIS and COST, two help programs of PHOENICS, we separately determined the length, width, and height, turbulence model, radiation model, grid division, and convergence residual of the computational domain. Referring to the measured data over the village and the perennial data on Weather Spark, we further determined the local weather parameters. Drawing on the standard for green performance calculation of civil buildings (JGJ/T 449-2018), we determined the wind profile function and its values. In addition, the independence and rationality of the grid size was tested by gradually increasing the number and density of grids. The increase was terminated, when the calculation result did not change significantly anymore.

#### 2.2.4. Parameter Setting for Heat Environment

The simulation parameters of the heat environment were configured similarly as those of the wind environment. In addition, the material parameters of the underlying surface, emission and absorption coefficients of solar radiation, and direct and diffuse solar radiations were determined, according to the standard for green performance calculation of civil buildings (JGJ/T 449-2018), code for thermal design of the civil building (GB 50176-2016), and local specifications. The common data are detailed in Tables 3 and 4.

#### 2.2.5. Parameter Setting for Green Plant Simulation

Green plants, which are usually porous media, should be modeled separately in Revit or Rhino, and imported to PHOENICS for converting to the Foliage type. The leaf area index, i.e., the ratio of the total area of plant leaves to the unit land area, was determined based on the actual physical characteristics. The drag coefficient is usually 0.15∼0.25 for deciduous trees, 0.2 for forests, 0.5 for a single row of deciduous trees, and 0.6∼1.2 for coniferous trees. The turbulence medication was set to green.  Table 5 presents the common plant parameters of traditional villages.

#### 2.2.6. Correlation Test

The Pearson correlation coefficient of the paired sample *t*-test is often adopted to measure the correlation between two variables. The value of the coefficient falls between −1 and 1. We corrected the parameters through the simulation of the village environment, and captured their values at an interval of 5 min. The simulation accuracy meets the requirement, only if the simulation value does not significantly vary from the measured value at any point (*P* > 0.05) [18]. Otherwise, at least one item in the simulation went wrong, and another round of simulation should be performed.

### 2.3. Composite Evaluation and Optimization Design

#### 2.3.1. Year-Round Climate Simulation

Based on the perennial data on Weather Spark (https://zh.weatherspark.com/), each year was divided into a comfort domain, a discomfort domain, and a transitional domain. Among them, the comfort domain refers to the natural days that are sufficiently comfortable, without needing any spatial optimization; the discomfort domain refers to the natural days that are not sufficiently comfortable, despite going through spatial optimization; the transitional domain refers to the natural days that are not yet sufficiently comfortable, but will meet the comfort requirement after spatial optimization. The spatial optimization is the process of improving the comfort level of spatial nodes in the transitional domain from discomfortable to comfortable.

In the field of Extenics, two intervals are often available to measure the satisfactoriness of the value of a feature in the domain of discourse *U*: the satisfactory interval *χ*_0_=〈*a*_0_,  *b*_0_〉, and the acceptable interval *x*=〈*a*,  *b*〉. It is clear that *X*⊃*X*_0_.

When no transform is implemented, if the value of the object on a feature falls in the acceptable interval 〈*a*,  *b*〉, then the object has a certain attribute. The degree for the object to have the attribute can be characterized by a real number in (0,  +*∞*). Such objects constitute the positive domain in the extension set. On the contrary, if the value of the object on a feature falls outside the acceptable interval 〈*a*,  *b*〉, then the object does not have the certain attribute. The degree for the object to lack the attribute can be characterized by a real number in (−*∞*, 0). Such objects constitute the negative domain in the extension set. If the value of the object on a feature is *a* or *b*, then the object is the zero boundary in the extension set.

The satisfactory interval *χ*_0_=〈*a*_0_,  *b*_0_〉 is the standard positive domain, which corresponds to the comfort domain; the interval *X*_+_=〈*a*,  *a*_0_〉 ∪ 〈*b*_0_,  *b*〉 is the transitional positive domain [25].

Similarly, the negative domain can be divided into a transitional negative domain, and a standard negative domain.

Let ℜ denote the real number domain, and *X*_−_=〈*c*,  *a*〉 ∪ 〈*b*,  *d*〉 denote the transitional negative domain. Suppose *X*^∧^=*X* ∪ *X*_−_=〈*c*,  *d*〉, the values of the negative domain fall in the interval *X*^−^=*R* − *X*, and the values of the standard negative domain fall in the interval of *X*_0_^−^=*R* − *X*^−^. Then, the domain of discourse *U* can be divided into the following:

(1) $$\begin{array}{c} \text{Domain of discourse }U\left\{\begin{array}{c} \text{Positive domain}\left\{\begin{array}{c} \text{Standard positive domain}\\ \text{Transitional positive domain} \end{array}\right.\\ \text{Zero boundary}\\ \text{Negative domain}\left\{\begin{array}{c} \text{Standard negative domain}\\ \text{Transitional negative domain} \end{array}\right. \end{array}\right.\text{.} \end{array}$$

In this study, the transitional positive domain and the transitional negative domain of Extenics are combined into the transitional domain, which precisely corresponds to the transitional domain of microclimate comfort. Based on the perennial data on Weather Spark, we determined four critical weather parameters of village microclimate, namely, *V*_cold(Winter⟶Spring)_, *V*_hot(Summer⟶Autumn)_, *V*_hot(Spring⟶Summer)_, and *V*_cold(Autumn⟶Winter)_ (Figure 5). The weather parameters include wind velocity, wind speed, outdoor air temperature, relative humidity, soil temperature at −3.2 m, intensity of direct solar radiation, and intensity of diffuse solar radiation.

#### 2.3.2. Preliminary Spatial Design

Spatial design adjusts and optimizes the design elements of the traditional village square through addition, deletion, and replacement, aiming to formulate a new design scheme. The design elements belong to such types of points, lines, surfaces, and masses. Among them, points and lines have a negligible impact on the microclimate. As an important feature of design elements, the material has a major impact on the simulation of the heat environment. Therefore, this study extracts, classifies, and grades the design elements in various excellent design cases similar to our project, considering the types of horizontal plane, vertical plane, mass, and material. In this way, a complete list of design elements was prepared for traditional village squares (Table 6).

#### 2.3.3. Wind Comfort Indices and Evaluation

Based on the influence of microclimate comfort on behaviors, the activities on the square are either static or dynamic. The static behaviors include sitting, chatting, and playing cards; the dynamic behaviors include recreation and sports activities, such as roller-skating, dancing, and working out. Considering the Beaufort wind comfort criteria, as well as the age and the activity type of different users in different seasons [19], this study takes 5 m/s as the maximum comfortable wind velocity, and defines the comfort level of different wind velocities: 0∼0.5 m/s (level 0), 0.5∼1 m/s (level 1), 1∼1.5 m/s (level 2), 1.5∼2 m/s (level 3), 2∼2.5 m/s (level 4), 2.5∼3 m/s (level 5), 3∼3.5 m/s (level 6), 3.5∼4 m/s (level 7), 4∼4.5 m/s (level 8), and 4.5∼5 m/s (level 9). These levels were defined by the INFORM function of PHOENICS, and recorded as LAWS (Table 7).

#### 2.3.4. Heat Comfort Indices and Evaluation

The UTCI, which comprehensively considers the spatiotemporal distribution of microclimate elements like wind, heat, humidity, and solar radiation, applies to the evaluation of the outdoor heat environment [20]. Thus, the study takes UTCI as the indicator of heat comfort [21]. The evaluation criteria are recorded in Table 8. The comfortable interval (no heat stress) is equivalent to the temperature range of 9°C∼26°C, and recorded as level 6. The temperature range of 0°C∼9°C is recorded as level 5. The rest can be obtained by analogy.

#### 2.3.5. Composite Comfort Evaluation

The wind and heat comfort was compositely evaluated by the composite correlation function. Let *λ*_1_, *λ*_2_,…, *λ*_*m*_ be the weight coefficients of microclimate features *c*_1_, *c*_2_,…, *c*_*m*_, and satisfy ∑_*i*=1_^*m*^*λ*_*i*_=1. The composite correlation [25] can be calculated by

(2) $$\begin{array}{c} K\left(B\right)=\sum_{i=1}^{m}\lambda_{i}k_{i}\left(c_{i}\left(B\right)\right)=\sum_{i=1}^{m}\lambda_{i}k_{i}\left(x_{i}\right). \end{array}$$

Before the calculation, all features must be normalized to the SME value range. Then, the experts of urban-rural planning and architecture were invited to determine the weights of wind and heat comfort. Expert surveys found that for ordinary traditional villages, the weights of wind and heat comfort are both equal to 0.5. Finally, the result was calculated by the INFORM function of PHOENICS, and recorded as COMF.

#### 2.3.6. Generation of Final Design Scheme

The preliminary design scheme was adjusted continuously according to the microclimate evaluation results. The scheme was viewed as the final design scheme, when the following condition was fulfilled: in the transitional domain, the microclimate comfort of the design scheme meets the requirements of all types of dynamic and static behaviors, and satisfies the physiological and psychological requirements of villagers and tourists; the modified design elements have practical functions and aesthetic beauty. As a key component of the village design, the final design scheme would contribute immensely to the future development of the village.

## 3. Case Analysis

The feasibility of our strategy was demonstrated with Xieduqi square, Zoumatang village, eastern China's Zhejiang Province as the example. Founded more than 1,000 years ago, the village is encircled by several rivers, making it a typical water town in the lower reaches of the Yangtze river. Over the history, 76 villagers received the title of Jinshi, the highest and final degree in the imperial examination in Imperial China. Therefore, the village is hailed as the largest cradle of Jinshi in China, and recognized as the famous Chinese historical and cultural village, and Chinese traditional village. It is located at the center of the village, the Xieduqi square was originally an artificially excavated river channel. The square gets its name for the 30 m-long oval pier next to the river channel, which looks like the belly button of a crab (the literal meaning of Xieduqi). The square is surrounded by 1-2 story ancient buildings in the style of eastern Zhejiang. The main streets run from east to west. On the river bank lies a long pavilion for tourists and residents to rest temporarily (Figure 6).

**Step 1 .**

Field measurement of wind and heat environments

The wind and heat environments were measured from 9am to 5pm on December 25^th^, 2020, using five ultrasonic integrated weather stations. One ultrasonic integrated weather station was placed at 1.5 m above the tallest building in the village, with no occlusions in the surroundings. The other four stations were, respectively, deployed inside the long pavilion, beneath the ancient tree, at the east entrance of the square, and at the west entrance of the square (Figures 7–9).

**Step 2 .**

Simulation of wind and heat environments

Referring to the simulation method in Section 2.2, the wind and heat environments at each measuring point of the square were simulated based on the weather parameters on December 25^th^, 2020. The simulation results are displayed in Figure 10 and Table 9.

**Step 3 .**

Comparison between simulation results and measured results

**Step 4 .**

Perform composite evaluation and optimization design

Through a year-round simulation of the Xieduqi square, it was learned that the wind velocity is small in summer due to the occlusion by the 1–2 story buildings on the south. In winter, the north wind is not effectively blocked, making it difficult to carry out static activities in the long pavilion. To solve these two problems, we provided a spatial optimization strategy for the square: (1) the village committee needs to buy back the two residential buildings on the south of the square, which are not inhabited for a long time and are inconsistent in style with the surroundings, at a reasonable price, and transform them into lawns; (2) a skylight needs to be opened on the top of the long pavilion, and provided with sun blinds that can be opened or closed at any time; (3) to block wind in winter, a transparent windscreen needs to be arranged on the northside in the long pavilion, which can be opened or closed at any time; (4) a winter outdoor activity area needs to be designed to the north of the long pavilion, and provided with temporary furniture (Figure 11).

The location and area of the skylight and windscreen will be adjusted constantly according to simulation results. None of these renovations affect the ancient buildings, historical landscapes, or related structures. All renovation measures target the newly built elements.

The microclimate comfort of the renovation scheme was simulated and evaluated. Figures 12 and 13 show the wind velocity, wind comfort, UTCI, and composite comfort of the scheme, facing the critical weather condition *V*_hot(Spring⟶Summer)_ in the transitional domain from spring to summer.

As shown in Figure 12, the additional lawns significantly accelerate the wind velocity on the square in summer. The wind moved faster than 1 m/s at any node in the key space for dynamic and static behaviors. The fast wind could carry away a huge amount of heat. Besides, these nodes had high wind comfort.

As shown in Figure 13, after continuous adjustments, the UTCI of any space in the square was smaller than 32°C, corresponding to the level of moderate heat stress. That is, the outdoor activities have a high heat comfort. For the main areas of the square, composite comfort was always above 1.5. The most comfortable state appeared inside and on the north of the long pavilion. Frequent recreation, entertainment, and ancient village experience activities can be arranged in these areas.

## 4. Conclusions

The evaluation and optimization design for microclimate comfort of traditional village squares based on extension correlation function make full use of digital technologies like oblique photography, panoramic shooting, and information modeling, and generate the optimization design scheme for traditional village squares through the following steps: field measurement of wind and heat environments, simulation of wind and heat environments, preliminary design of microclimate comfort, and composite evaluation of microclimate comfort.

1. In order to realize year-round climate simulation, the four critical weather parameters of traditional villages in a certain area can be determined by using the “transition domain” in the extension correlation function and the weather data of the Weather Spark website over the years. They were recorded as *V*_cold(Winter⟶Spring)_, *V*_hot(Summer⟶Autumn)_, *V*_hot(Spring⟶Summer)_, and *V*_cold(Autumn⟶Winter)_.
2. A series of parameter values were determined in microclimate comfort simulation, including the length, width, and height of the calculation area, turbulence model, discretization equation, radiation model, grid division, convergence residual, solar absorption and radiation coefficient, plant leaf area index, and drag index.
3. Wind comfort (LAWS), with 5 m/s as the limit value, was divided into 10 levels, and established the corresponding relationship between wind speed and season, and user age and the activity type. According to −40°C, −27°C, −13°C, 0°C, 9°C, 26°C, 32°C, 38°C, and 46°C, heat comfort (UTCI) was divided into 10 levels, and the comfort zone (i e, no thermal stress) was from 9°C to 26°C.
4. A comprehensive evaluation method of microclimate comfort in traditional village was proposed, based on the comprehensive correlation function and the inform function of PHOENICS. Wind and heat comfort must be normalized to the SME value range, and their weights are both equal to 0.5.
5. A digital technology system for evaluating micro-climate comfort in traditional villages has been established. The relevant software and hardware were drone (DJI Phantom 4 pro v2.0), DJI pilot, ContextCapture, Panoramic Camera (Insta360 Pro 2), Revit, Dynamo, Rhino, PHOENICS, and ultrasonic integrated weather station (RS-FSXCS-N01-1).

The following work will be implemented in the future:

1. To determine the weight of wind and heat comfort for traditional villages with special comfort evaluation needs;
2. To explore methods for establishing traditional village information models more quickly, automatically, and in batches;
3. To expand to the method of microclimate comfort evaluation of traditional village streets, courtyards, and indoor spaces of public buildings.

## Figures and Tables

**Figure 1:** Flow of evaluation and optimization design.

**Figure 2:** Cloud platform.

**Figure 3:** Aerial model.

**Figure 4:** Information model.

**Figure 5:** Year-round climate division.

**Figure 6:** The current situation of the Xieduqi square. (a) Looking from the west. (b) Looking from the east.

**Figure 7:** Measured weather parameters of the Zoumatang village.

**Figure 8:** General plan of the Xieduqi square.

**Figure 9:** Location of ultrasonic integrated weather stations. (a) Measuring point 1. (b) Measuring point 2. (c) Measuring point 3. (d) Measuring point 4.

**Figure 10:** Simulated environments of the Xieduqi square. (a) Wind velocity. (b) Temperature.

**Figure 11:** Optimization design strategy for the square.

**Figure 12:** Simulation results for the optimal design scheme of the square (part 1). (a) Wind velocity. (b) Wind comfort.

**Figure 13:** Simulation results for the optimal design scheme of the square (part 2). (a) UTCI. (b) Composite comfort.

**Table 1:** Summary of relevant review studies on microclimate comfort.

No.	Author	Year	Ref.	Field measurement	Year-round climate	Wind comfort	Heat comfort	The behaviors
1	Sodoudi et al	2018	[1]				●	
2	Tsoka et al	2018	[2]				●	
3	Wu et al	2019	[3]				●	
4	Aldeek	2020	[4]		●		●	
5	Teshnehdel et al	2020	[5]				●	
6	Middel et al	2014	[6]				●	
7	Galal et al	2020	[7]	●			●	
8	Forouzandeh	2018	[8]	●			●	
9	López-Cabeza et al	2018	[9]	●			●	
10	Tumini et al	2016	[10]	●			●	
11	Chatzidimitriou, Yannas	2016	[11]				●	
12	QIU, Yu	2021	[12]				●	
13	Huang	2016	[13]			●		●
14	Yan et al.	2020	[14]		●		●	●
15	Gaspari, Fabbri	2017	[15]				●	
16	Zaki et al	2020	[16]	●			●	
17	Fabbri, Costanzo	2020	[17]	●				
18	Chan, Chau	2021	[18]	●			●	
19	Graham et al	2020	[19]				●	
20	Kamel	2021	[20]				●	
21	Potchter et al	2022	[21]				●	

**Table 2:** Initial technical parameters.

Range	Starting wind velocity	0.01 m/s
	Wind velocity	0∼60 m/s
	Wind direction	0∼359°
	Humidity	0% RH∼99% RH
	Temperature	−40°C∼+80°C
	Atmospheric pressure	0∼120 kPa

Precision	Wind velocity	±(0.2 m/s ± 0.02^*∗*^*v*) (*v* is the real wind velocity)
	Wind direction	±3°
	Humidity	±3% RH (60% RH, 25°C)
	Temperature	±0.5°C (25°C)
	Atmospheric pressure	±0.15 kPa@25°C 75 kPa

Resolution	Wind velocity	0.01 m/s
	Wind direction	1°
	Humidity	0.1% RH
	Temperature	0.1°C
	Atmospheric pressure	0.1 kPa

**Table 3:** Setting of environment simulation parameters.

Parameter	Input
Latitude	Latitude of the village (29.72°N for Zoumatang village)
Turbulence model	RANS *k* – *ε* (close to the result of wind tunnel test [28])
Discretization equation	Simple, PRESTOL
Wind profile function	Wind velocities obeying exponential distribution, *α* = 0.16
Radiation model	IMMERSOL
Computational domain	On the edge of building(s), the boundary of the computational domain is 7 times of the height H of the building in the horizontal direction, and 6 times of H in the vertical direction. Hence, the windward profile blocking rate is smaller than 3%.
Grid division	There are no fewer than 5 grids in the space 1.5 m above the ground; the grid expansion rate is 1.2; grid independence is verified.
Convergence residual	The residue is within 10^−4^; the imbalance of the equation is within 1%; the value of the representative monitoring points in the flow field does not change or fluctuates about a fixed value.
Direct solar radiation	Following the code for thermal design of the civil building (GB 50176-2016), or local specifications
Diffuse solar radiation	

Air temperature	Referring to the measured data over the village and the perennial data on Weather Spark
Wind velocity (*h* = 10 m)	
Wind direction	
Relative humidity	
Temperature	
Air pressure	

**Table 4:** Emission and absorption coefficients of solar radiation.

Component	Material	Surface attribute	Color	Emissivity	Absorptivity
Roof	Reddish brown clay tile roof	Old	Reddish brown	0.85∼0.95	0.65∼0.74
	Gray tile roof	Old	Light gray	0.85∼0.95	0.52

Wall	Lime powder wall	Smooth and new	White	0.85∼0.95	0.48
Water body	Silicate brick wall	Unsmooth	Red	0.85∼0.95	0.50
	Water (lake, and sea surface)	—	—	0.95∼0.99	0.96

Vegetation	Green grass	—	—	0.97∼0.99	0.78∼0.80
	Permeable brick	—	—	0.85∼0.95	0.74
	Grow-through paver	—	—	0.85∼0.95	0.74

Road and square	Ordinary cement	—	Gray	0.85∼0.95	0.74
	Asphalt pavement	—	Dark gray	0.9	0.87
	Soil	—	—	0.9	0.80

**Table 5:** Common plant parameters.

Type of plant	Leaf area index	Drag coefficient	*C*_*pe1*_	*C*_*pe2*_	Emissivity	Absorptivity
Mixed broadleaf-conifer forest	3	0.5	1.8	0.6	0.98	0.8
Grassland with sparse trees	2	0.2	1.8	0.6	0.98	0.8
Lawn	4	0.045	1.8	0.6	0.98	0.8
Arbor	3	0.5	1.8	0.6	0.98	0.8
Camphor	5.5	0.5	1.8	0.6	0.98	0.8
Magnolia	6.5	0.5	1.8	0.6	0.98	0.8

**Table 6:** Complete list of design elements was prepared for traditional village squares.

Type	Design form	Design element
Horizontal plane	Ground	Wooden platform, bridge, water surface, road, pavement, etc.
	Ground	Pavilion, shed, corridor, eaves, tree crown, parasol, etc.

Vertical plane	Independent wall	The wall has openings, or can be turned into doors through overall transformation; tile wall, gabion wall, tree array, etc.
	*L*-shaped wall	
	Parallel walls	
	*U*-shaped wall	
	Enclosed walls	

Mass		The whole building is newly constructed or demolished; morphological changes
Material	Wall	Loam, colored drawing, glass, wooden board, red brick, gray brick, white plaster, bluestone, etc.
	Ground	Soil, asphalt concrete; permeable brick, planted vegetation; wooden board; water surfaces like lake, pond, and river; stones like granite and pebble.
	Roof	Thatch, wooden board, red tile, brown tile, gray tile, etc.

**Table 7:** Comfort levels of wind environment on the square.

Type of activity	Name of activity	Group	Comfort level (summer)	Comfort level (winter)
Sitting activities	Playing cards	Seniors	0∼1	0
	Resting and chatting	—	2	1

Standing activities	Taking photos, reading bulletins, and sightseeing	—	3	2
Walking activities	Strolling, and walking dogs	—	4	3
Recreation and sports activities	Children's entertainment activities	Children	5	4
	Shadow boxing, and sword dancing	Seniors	6	5
	Flying a kite	Seniors	7	6
	Skating, running, working out, and dancing	—	8	7

Passing through	—	—	9	8

**Table 8:** UTCI levels.

UTCI (°C)	Physiological stress level
>46	Extreme heat stress
38 to 46	Very strong heat stress
32 to 38	Strong heat stress
26 to 32	Moderate heat stress
9 to 26	No heat stress
0 to 9	Slight cold stress
−13 to 0	Moderate cold stress
−27 to −13	Strong cold stress
−40 to −27	Very strong cold stress
<−40	Extreme cold stress

**Table 9:** Measured values at each measuring point of the square.

Time series	Measuring point 1		Measuring point 2		Measuring point 3		Measuring point 4	
Node name	Wind velocity (m/s)	Temperature (°C)	Wind velocity (m/s)	Temperature (°C)	Wind velocity (m/s)	Temperature (°C)	Wind velocity (m/s)	Temperature (°C)
09-10	0.95	5.00	0.58	4.86	0.43	5.53	0.89	4.94
10-11	0.86	4.65	0.76	4.40	0.50	5.18	0.75	4.32
11-12	0.80	4.50	0.76	4.27	0.51	5.01	0.65	4.30
12-13	0.94	4.51	0.73	4.31	0.44	5.08	0.90	4.50
13-14	0.83	4.32	0.70	4.09	0.41	4.83	0.78	4.52
14-15	0.47	3.98	0.50	3.75	0.42	4.52	0.54	3.95
15-16	0.86	4.14	0.78	3.92	0.51	4.59	0.84	4.20
16-17	0.83	4.06	0.89	3.85	0.43	4.48	0.81	3.92

**Table 10:** Simulation results at each measuring point of the square.

Time series	Measuring point 1		Measuring point 2		Measuring point 3		Measuring point 4	
Node name	Wind velocity (m/s)	Temperature (°C)	Wind velocity (m/s)	Temperature (°C)	Node name	Wind velocity (m/s)	Temperature (°C)	Wind velocity (m/s)
09-10	0.82	4.80	0.50	4.52	0.38	5.42	0.81	4.64
10-11	0.79	4.25	0.66	4.24	0.47	5.03	0.69	4.01
11-12	0.90	4.30	0.71	4.01	0.47	4.88	0.61	4.23
12-13	0.87	4.29	0.63	4.03	0.42	5.21	0.87	4.13
13-14	0.90	4.12	0.61	3.88	0.39	4.76	0.72	4.29
14-15	0.41	3.72	0.42	3.26	0.38	4.32	0.44	3.83
15-16	0.81	4.00	0.67	3.67	0.56	4.44	0.79	4.15
16-17	0.75	4.13	0.79	3.77	0.45	4.38	0.76	3.80

**Table 11:** Fitness between simulation and measured results at each measuring point of the square.

	Measuring point 1		Measuring point 2		Measuring point 3		Measuring point 4	
	Wind velocity (m/s)	Temperature (°C)	Wind velocity (m/s)	Temperature (°C)	Node name	Wind velocity (m/s)	Temperature (°C)	Wind velocity (m/s)
Equation	*y* = *a* + *b*^*∗*^*x*	*y* = *a* + *b*^*∗*^*x*	*y* = *a* + *b*^*∗*^*x*	*y* = *a* + *b*^*∗*^*x*	*y* = *a* + *b*^*∗*^*x*	*y* = *a* + *b*^*∗*^*x*	*y* = *a* + *b*^*∗*^*x*	*y* = *a* + *b*^*∗*^*x*
Weight	Unweighted	Unweighted	Unweighted	Unweighted	Unweighted	Unweighted	Unweighted	Unweighted
Intercept	0.02563 ± 0.17626	0.53378 ± 0.62552	−0.05218 ± 0.04303	−0.24668 ± 0.58233	−0.11303 ± 0.14426	−0.45755 ± 0.52582	−0.12729 ± 0.05036	0.82598 ± 0.50074
Slope	0.92431 ± 0.2125	0.83446 ± 0.14195	0.94867 ± 0.05964	0.99711 ± 0.13882	1.21212 ± 0.31498	1.07344 ± 0.10699	1.08902 ± 0.06468	0.76399 ± 0.11532
Residual sum of squares	0.04268	0.09798	0.00221	0.10468	0.00761	0.06467	0.00265	0.06124
Pearson's R	0.87134	0.92307	0.98835	0.94647	0.8436	0.97147	0.98958	0.93794
*R* ^2^ (COD)	0.75923	0.85206	0.97684	0.89581	0.71166	0.94374	0.97927	0.87974
Adjusted *R*^2^	0.71911	0.8274	0.97298	0.87845	0.66361	0.93437	0.97582	0.8597

The simulated results were fitted against the measured results through the paired sample *t*-test. The results show that the *R*^2^ at any measuring point was greater than 0.5, a sign of strong correlation. There is no significant difference between the two sets of results (*P* > 0.05), i.e., the simulation is sufficiently accurate (Tables 10 and 11).

## Data Availability

The data used to support the findings of this study are available from the corresponding author upon request.
